The article "In vitro and in vivo anti-colon cancer effects of Garcinia mangostana xanthones extract" was retracted in 2022. Reasons: ethical violations by an author; concerns about the data.

# *In vitro and in vivo anti-colon cancer effects of Garcinia mangostana* xanthones extract

**DOI:** 10.1186/1472-6882-12-104

**Published:** 2012-07-20

**Authors:** Abdalrahim F A Aisha, Khalid M Abu-Salah, Zhari Ismail, Amin Malik Shah Abdul Majid

**Affiliations:** 1 Department of Pharmacology, School of Pharmaceutical Sciences, Universiti Sains Malaysia, Minden, 11800, Pulau Penang, Malaysia; 2 The Chair of Cancer Targeting and Treatment, Biochemistry Department and King Abdullah Institute for Nanotechnology, King Saud University, Riyadh, 11451, Saudi Arabia; 3 Department of Pharmaceutical Chemistry, School of Pharmaceutical Sciences, Universiti Sains Malaysia, Minden, 11800, Pulau Penang, Malaysia; 4 Australian Institute for Nanotechnology and Bioengineering, University of Queensland, Queensland, 4072, Australia

## Abstract

**Background:**

Xanthones are a group of oxygen-containing heterocyclic compounds with remarkable pharmacological effects such as anti-cancer, antioxidant, anti-inflammatory, and antimicrobial activities.

**Methods:**

A xanthones extract (81% α-mangostin and 16% γ-mangostin), was prepared by crystallization of a toluene extract of *G. mangostana* fruit rinds and was analyzed by LC-MS. Anti-colon cancer effect was investigated on HCT 116 human colorectal carcinoma cells including cytotoxicity, apoptosis, anti-tumorigenicity, and effect on cell signalling pathways. The *in vivo* anti-colon cancer activity was also investigated on subcutaneous tumors established in nude mice.

**Results:**

The extract showed potent cytotoxicity (median inhibitory concentration 6.5 ± 1.0 μg/ml), due to induction of the mitochondrial pathway of apoptosis. Three key steps in tumor metastasis including the cell migration, cell invasion and clonogenicity, were also inhibited. The extract and α-mangostin up-regulate the MAPK/ERK, c-Myc/Max, and p53 cell signalling pathways. The xanthones extract, when fed to nude mice, caused significant growth inhibition of the subcutaneous tumor of HCT 116 colorectal carcinoma cells.

**Conclusions:**

Our data suggest new mechanisms of action of α-mangostin and the *G. mangostana* xanthones, and suggest the xanthones extract of as a potential anti-colon cancer candidate.

## Background

*Garcinia mangostana* L. or mangosteen is a tropical tree from the family Clusiaceae. The tree is cultivated for centuries in Southeast Asia rainforests, and can be found in many countries worldwide [1]. Pericarps of the fruit have been used in folk medicine for the treatment of many human illnesses such as skin and wound infections, and inflammatory diseases [2]. Mangosteen is also used as an ingredient in several commercial products including nutritional supplements, herbal cosmetics, and pharmaceutical products [1].

The article "In vitro and in vivo anti-colon cancer effects of Garcinia mangostana xanthones extract" was retracted in 2022. Reasons: ethical violations by an author; concerns about the data.

Mangosteen fruit rinds contain high concentration of xanthones. α-Mangostin (1,3,6-trihydroxy-7-methoxy-2,8-bis(3-methyl-2-butenyl)-9 H-xanthen-9-one), and γ-mangostin (1,3,6,7-tetrahydroxy-2,8-bis(3-methylbut-2-enyl)xanthen-9-one) (Figure 1) are the main xanthones isolated from *G. mangostana*[3,4].

**Figure 1:** **Chemical structure of α-mangostin and γ-mangostin, the main constituents of the** ***G. mangostana*** **xanthones extract.**

The *G. mangostana* xanthones are gaining more and more interest due to their remarkable pharmacological effects including analgesic [5], antioxidant [6], anti-inflammatory [7], anti-cancer [8-11] anti-allergy [12], antibacterial [13], anti-tuberculosis [14], antifungal [15], antiviral [16], cardioprotective [17], neuroprotective [18], and immunomodulation [19] effects.

Colorectal cancer is the third in incidence after lung and breast cancers and accounts for almost 10% of total cases of cancer and almost 8% of total cancer deaths [20]. According to the World Health Organization (WHO), more than 70% of all cancer deaths occurred in countries with low and middle income, and deaths from cancer worldwide are projected to continue to rise to over 11 million in 2030 [21]. Hence, there is an increasing demand for cost-effective therapeutics and chemoprevention agents for the various types of cancer. Several studies have shown natural products, particularly medicinal plants as potential chemoprevention and anti-cancer candidates.

Anti-cancer properties of *G. mangostana* extracts or pure xanthones have been extensively studied *in vitro*, however few reports of *in vivo* anti-cancer effects could be traced. Xanthone extracts from *G. mangostana* have been reported with chemoprevention effects against the chemically induced colon cancer [8], suppression of tumor growth and metastasis in a mouse model of mammary cancer [9], and a recent report showed the inhibition of prostate cancer growth by α-mangostin, the main constituent of the *G. mangostana* xanthones [22].

This study aims to investigate the *in vitro* anti-colon cancer properties of a *G. mangostana* xanthones extract (81% α-mangostin and 16% γ-mangostin) on HCT 116 human colorectal carcinoma. The *in vitro* anti-cancer effects include cytotoxicity, apoptosis, cell migration, cell invasion, and clonogenicity. The mechanism of action of the xanthones extract and α-mangostin on the transcription factor level of 10 signalling pathways involved in colon carcinogenesis was also investigated. The study also aims to investigate the *in vivo* anti-colon cancer effect on a pre-established subcutaneous tumor of HCT 116 cells in NCR nude mice.

The article "In vitro and in vivo anti-colon cancer effects of Garcinia mangostana xanthones extract" was retracted in 2022. Reasons: ethical violations by an author; concerns about the data.

## Methods

### Cell lines and reagents

Human colorectal carcinoma cell line HCT 116; Catalogue number (CCL-247) and CCD-18Co normal colonic fibroblast; Catalogue number (CRL-1459) were purchased from the American Type Culture Collection (ATCC; Manassas, Virginia). RPMI 1640, Opti-MEM® and DMEM cell culture media, heat inactivated fetal bovine serum (HI-FBS), and phosphate buffered saline (PBS) without calcium and magnesium were purchased from Bio-Diagnostics (Petaling Jaya, Selangor, Malaysia). Cignal finder™ 10-pathway reporter-array system, and matrigel matrix (10 mg/ml) were purchased from SABiosciences (Frederick, Maryland). Wizard® SV genomic DNA purification system, caspases-3/7, -8 and −9 reagents, trans fast liposome, and dual luciferase reporter system were purchased from Promega (Petaling Jaya, Selangor, Malaysia). Cisplatin, Hoechst 33258, Rhodamine 123, agarose, ethidium bromide, penicillin/streptomycin (PS) solution, dimethylsulfoxide (DMSO), phenazine methosulfate (PMS), and 2,3-Bis(2-methoxy-4-nitro-5-sulfophenyl)-2 *H*-tetrazolium-5-carboxanilide inner salt (XTT) were purchased from Sigma-Aldrich (Kuala Lumpur, Malaysia). The solvents were of analytical or HPLC grade and were obtained from Avantor Performance Materials (Petaling Jaya, Selangor, Malaysia).

### Plant material and extraction

Ripened *G. mangostana* fruit was collected from a local fruit farm at Island of Penang, Malaysia. A voucher specimen (11155) was deposited at the Herbarium of School of Biological Sciences, USM. The fruit rind was chopped and dried at 45–50°C for 24 h. Toluene extract was prepared by maceration method at 1:5 plant: solvent ratio (wt/v), at 60°C for 48 h. The extract was filtered, concentrated at 60°C by rotavapor to about 150 ml, and crystallized at 2–8°C for 24 h. A yellow solid was formed, which was collected and dried at 50°C.

### Animals

Athymic NCR nu/nu nude mice were obtained from Taconic Farms Inc. (Hudson, New York). Mice were housed in specific pathogen free (SPF) cages supplied with high efficiency particulate air (HEPA) filters. Free access to autoclaved food and water was provided and the autoclaved bedding was changed twice weekly. The procedures were approved by the USM Animal Ethics Committee with a reference number PPSG/07(A)/044/(2010) (59).

### Liquid chromatography-mass spectrometry (LC-MS)

The xanthones extract was analyzed by a Dionex-Ultimate® 3000 Rapid Separation LC system (Dionex, Sunnyvale, California), connected with a Micro TOF-Q mass spectrometer (Bruker, Madison, Wisconsin). Chromatographic separation was performed using Nucleosil C18 column (5 μm, 4.6 × 250 mm) (Macherey-Nagel, Bethlehem, Pennsylvania), at 30°C, the mobile phase was consisting of 95% acetonitrile and 5% of 0.1% formic acid in water. The flow rate was set at 0.5 ml/min for 15 min, and spectral data were collected at 244 nm. Mass analysis was performed in the range 50–1000 m/z, under negative ion mode, and the nebulizer was set at 3.0 bar and heated to 150°C. The capillary voltage was set at 3000 V using a nitrogen dry gas at 8.0 L/min. The end plate offset was maintained at −500 V.

The article "In vitro and in vivo anti-colon cancer effects of Garcinia mangostana xanthones extract" was retracted in 2022. Reasons: ethical violations by an author; concerns about the data.

### Cell culture

HCT 116 cells were maintained in RPMI 1640 medium supplemented with 10% HI-FBS and 1% PS, and the CCD-18Co cells were maintained in DMEM medium supplemented with 10% HI-FBS and 1% PS. Cells were cultured in a 5% CO_2_ in a humidified atmosphere at 37°C.

### Cell viability

Cell viability was determined by the XTT test as described previously [23]. Briefly, cells were treated for 48 h, the culture medium was removed and replaced with a fresh one containing XTT and PMS at 100 μg/ml and 1 μg/ml, respectively. After incubation for 4 h, the optical density was measured at a wavelength of 450 nm, using a microplate reader (Thermo Fisher Scientific, Ratastie, Vantaa, Finland). The results are presented as a percentage inhibition to the negative control (0.5% DMSO) as the following:

(1) $$\text{Percentage inhibition}=(1–\frac{{\text{OD}}_{\text{Samples}}–{\text{ OD}}_{\text{Blank}}}{{\text{OD}}_{\text{Vehicle}}–{\text{ OD}}_{\text{Blank}}})\times 100$$

The median inhibitory concentrations (IC_50s_) were calculated from the dose response curves (n = 3).

### Caspases-3/7, -8 and −9

HCT 116 cells were treated in a white 96-well plate for 90 min. Subsequently, the caspases activity was measured by caspase Glo 3/7, Glo 8 and Glo 9 as described previously [24]. Luminescence was measured by a microplate reader (Hidex, Mustionkatu, Turku, Finland), and the results are presented as a mean of relative light units (RLU) ± SD (n = 4).

### Mitochondrial membrane potential and chromatin condensation

Rhodamine 123 and Hoechst 33258 were used as probes to study the effect on mitochondrial membrane potential and chromatin condensation [25,26]. Briefly, HCT 116 cells were treated with α-mangostin or the xanthones extract at different concentrations for 2 h. Subsequently, cells were fixed in 4% paraformaldehyde for 20 min, simultaneously stained with rhodamine 123 at 1 μg/ml and Hoechst 33258 at 10 μg/ml for 20 min, washed extensively with PBS, and examined immediately using IX71 inverted fluorescent microscopy (Olympus, Shinjuku, Tokyo, Japan). Cell morphology was evaluated by studying 5 randomly selected microscopic fields and the apoptotic index was calculated.

The article "In vitro and in vivo anti-colon cancer effects of Garcinia mangostana xanthones extract" was retracted in 2022. Reasons: ethical violations by an author; concerns about the data.

### DNA fragmentation

HCT 116 (2 × 10^6^) cells were treated for 48 h. Subsequently, the floating and attached cells were collected by centrifugation at 3000 rpm for 10 min, the total genomic DNA was extracted using Wizard® SV genomic DNA purification system, and analyzed by electrophoresis on 1.2% agarose gel stained with 0.5 μg/ml ethidium bromide.

### Anti-tumorigenicity

Anti-tumorigenicity studies including clonogenicity, cell migration, and cell invasion were investigated on HCT 116 cells. Effect on the clonogenicity was evaluated by the colony formation assay as previously described [27]. Five hundred cells were seeded in 6-well plate in 2.5 ml of RPMI 1640 medium, and were incubated to allow attachment. Subsequent to 48 h treatment, the drug was removed and cells were incubated in a fresh medium for 12 days. Colonies were fixed in 4% paraformaldehyde, stained with 0.5% crystal violet, and counted under a stereomicroscope. The plating efficiency (PE) of untreated cells and the survival fraction (SF) of treated cells were then determined (n = 3).

The effect on cell migration was studied by the wound healing assay as described previously [28]. Cell’s monolayer was scratched using a 200-μl micropipette tip, the detached cells were washed off, and the cells were treated in a medium containing 2% serum. The wounds were then photographed at zero time and incubated for 24 h. The distance of cell-free wounds was then measured using a Leica QWin image analysis software (Leica Microsystems Inc., Buffalo Grove, Illinois), and the percentage of wound closure was calculated relative to zero time.

Effect on cell invasion was studied by a modification of the Boyden chamber assay using matrigel matrix [29]. Basically, 50 μl of matrigel (5 mg/ml) was loaded into 96-well plate and allowed to solidify for 45 min. Treated cells (5 × 10^3^ in 150 μl RPMI medium) was added to each well and incubated for 48 h. Subsequently, cells were washed with PBS and the number of the invading cells was determined under inverted light microscopy. The results are presented as a percentage inhibition to untreated cells (n = 3).

### Effect on cell signalling pathways

The assay was performed in 96-well plate format according to the manufacturer’s instructions. Briefly, HCT 116 cells were transfected by reverse transfection with DNA constructs of 10 signalling pathways, a positive control, and a negative control. After overnight incubation, cells were treated for 6 h in complete RPMI medium. Subsequently, the activity of Firefly and *Renilla* luciferases was measured using dual-luciferase assay. The results are displayed as relative luciferase units, generated by dividing the Firefly/*Renilla* ratio of transcription factor-responsive reporter transfections by the Firefly/*Renilla* ratio of negative control transfections (n = 3). The fold change in the transcription factor activity was then calculated by dividing the results of the treated cells by that of untreated cells.

The article "In vitro and in vivo anti-colon cancer effects of Garcinia mangostana xanthones extract" was retracted in 2022. Reasons: ethical violations by an author; concerns about the data.

### *In Vivo* anti-tumor activity

Twenty four nude mice aged 6–8 weeks with average weight of 25 g were injected subcutaneously in right flank with 5 × 10^6^ cells in 150 μl RPMI. After 7–10 days, animals with uniform tumor size were divided into 3 groups of 6 animals. Tumor size and body weight were recorded before starting the treatment and at 5-days intervals for 20 days. Animals were treated by mixing the extract with the animal food at 0.25% and 0.5% extract: food ratio (wt/wt). Tumor dimensions were measured by a calibre in 2 angles, length and width [30]. Tumor size was then calculated as described previously [30-32], by applying the formula (((W + L)/2) ^ 3) × 2, where W is the width and L is the length. Tumor size in tumors with more than a lobe was calculated by summation of the size of the individual lobes [30]. Cross sections of the tumors were then prepared, stained with Eosin/Hematoxylin, and were studied for presence of necrotic cells and for the number of intratumor blood vessels. Blood vessels were counted at 20× magnification in 25 microscopic fields per tumor, and the results are presented as average number of blood vessels per tumor ± SD.

### Statistical analysis

The results are presented as mean ± SD. The differences between groups were compared by One-way ANOVA, and were considered significant at P < 0.05. Data analysis was carried out using SSPS 16.0 software.

## Results

### Phytochemical analysis

The extract was obtained at 5% yield (wt/wt) relative to the dry plant material. LC-MS analysis indicates the presence of 5 compounds; α-mangostin, was 81%, γ-mangostin was 16%, and the other 3 compounds were 3%, the percentage of the compounds was calculated based on the peak area (Table 1).

**Table 1:** **Mass spectrometry of the** ***G. mangostana*** **xanthones extract**

**Peak No**	**Retention time (min)**	**% Intensity**	**Isotopic pattern [M-H]- (m/z)**	**Molecular formula**	**Compounds**
1	7.4 ± 0.006	1.4 ± 0.1	413.1408	C_23_H_26_O_7_	Garcinone C
			414.1443		
			415.1397		
2	7.8 ± 0.001	15.6 ± 1.6	395.1308	C_23_H_24_O_6_	γ-mangostin
			396.1338		
			397.1360		
3	8.8 ± 0.013	1.2 ± 0.1	379.1370	C_23_H_24_O_5_	8-deoxygartanin
			380.1381		
			381.1440		
4	9.2 ± 0.001	80.8 ± 1.6	409.1452	C_24_H_26_O_6_	α-mangostin
			410.1489		
			411.1526		
5	13.5 ± 0.005	0.9 ± 0.03	423.1604	C_25_H_28_O_6_	β-mangostin
			424.1631		
			425.1667		

The mass was recorded in the negative ion mode (n = 4).

The article "In vitro and in vivo anti-colon cancer effects of Garcinia mangostana xanthones extract" was retracted in 2022. Reasons: ethical violations by an author; concerns about the data.

### Cytotoxicity

The xanthones extract, α-mangostin, and γ-mangostin caused dose dependent killing of the colon cancer cells (Figure 2a), showing IC_50s_ of 6.5 ± 1.0 μg/ml, 5.1 ± 0.2 μg/ml, and 7.2 ± 0.4 μg/ml, respectively. CCD-18Co normal cells, unlike HCT 116 cells, were 2 folds less sensitive showing IC_50_ of 11.1 ± 0.4 μg/ml (α-mangostin), and 13.0 ± 0.6 μg/ml (xanthones extract). Cisplatin, as a positive control, also showed dose dependent cytotoxicity on colon cancer cells giving IC_50_ of 6.1 ± 0.2 μg/ml.

**Figure 2:** **Cytotoxic and apoptotic effects of α-mangostin and the xanthones extract on HCT 116 cells.** Dose response curves of the xanthones extract on HCT 116 and CCD-18Co cells in the concentration range 2.5 – 30 μg/ml (a). Effect on caspases-3/7 (b), and caspases-8 and −9 (c). Effect on DNA fragmentation (d): the negative control was 0.5% DMSO, the positive control was α-mangostin at 20 μg/ml, and the xanthones extract was applied at 10, 20, 30 and 40 μg/ml. (*) indicates *P* < 0.05.

### Effect on caspases-3/7,-8 and −9

α-Mangostin and the xanthones extract at 10 and 20 μg/ml, showed a rapid enhancement of the caspases-3/7 activity after a treatment for 90 min (Figure 2b). At a concentration of 5 μg/ml, a slight but not significant increase in the activity was achieved (P > 0.05). The treatment compounds also caused significant enhancement of the caspase-9 activity in HCT 116 cells, but not caspase-8 activity (Figure 2c). The increase in caspase-9 activity was almost 8-folds more than that of caspase-8.

### Effect on DNA fragmentation

Analysis of the total genomic DNA by agarose gel electrophoresis revealed apparent DNA fragmentation in HCT 116 cells (Figure 2d). The results indicate that the effector caspases executed the apoptotic signal stimulated by the treatment compounds.

### Effect on mitochondrial membrane potential of HCT 116 cells

The rhodamine staining showed a distinct morphology of the apoptotic cells, which were stained more brightly than the non-apoptotic cells (Figure 3a). The result indicates lower concentration of rhodamine 123 due to loss of mitochondrial membrane potential. The apoptotic index of α-mangostin-treated cells at 20 μg/ml was (55 ± 9)%, and that of the xanthones extract was (13.2 ± 2.4)%, (38 ± 4.5)%, (47 ± 4.5)%, and (68 ± 9)% at 7.5, 10, 15 and 20 μg/ml, respectively. Significant induction of apoptosis, compared to untreated cells (5.1 ± 2.3)%, was obtained at the last 3 concentrations (P = 0.0), whereas no significant effect was observed at a concentration of 7.5 μg/ml (P = 0.2).

**Figure 3:** **Effect the xanthones extracts on mitochondrial membrane potential and chromatin condensation.** The mitochondrial membrane potential (a): negative control (1), α-mangostin at 20 μg/ml (2) and the xanthones extract at 20 μg/ml (3). Chromatin condensation (b): negative control (1), α-mangostin at 20 μg/ml (2) and the xanthones extract at 20 μg/ml (3).

The article "In vitro and in vivo anti-colon cancer effects of Garcinia mangostana xanthones extract" was retracted in 2022. Reasons: ethical violations by an author; concerns about the data.

### Effect on chromatin condensation and nuclear fragmentation

α-Mangostin at 20 μg/ml, and the xanthones extract caused significant and dose dependent induction of chromatin condensation and nuclear fragmentation in HCT 116 cells after 2 h treatment. Staining with the DNA probe Hoechst 33258 produced a distinct nuclear morphology of the apoptotic cells, which were stained more brightly, with or without nuclear fragmentation, whereas the non-apoptotic cells showed uniformly stained nuclei at lower intensely (Figure 3b). The apoptotic index of α-mangostin-treated cells was (47 ± 5.5)%, and that of the extract was (4.4 ± 3)%, (37 ± 7)%, (39 ± 10)%, and (52 ± 9)% at 7.5, 10, 15 and 20 μg/ml, respectively. Compared with the vehicle alone (3.3 ± 3)%, significant induction of apoptosis was obtained at 10, 15 and 20 μg/ml (P = 0.0), whereas the treatment at 7.5 μg/ml did not show any apoptotic effect, (P = 0.99).

### Anti-tumorigenicity

The compounds inhibited the clonogenicity of HCT 116 cells (Figure 4a). The PE was (54 ± 2)%, and the SF in cells treated with the xanthones extract was 0% at all concentrations. The SF in α-mangostin treated cells was 0% at 20, 15, 10 and 7.5 μg/ml, and (7.8 ± 0.3)% at 5 μg/ml.

**Figure 4:** **Anti-tumorigenicity effect of the xanthones extract on HCT 116 cells.** Clonogenicity (a): negative control (1), α-mangostin at 5 μg/ml (2) and the xanthones extract at 5 μg/ml (3). Cell migration (b): wounds photographed at zero time (1), and the treated cells after 24 h; negative control (2), α-mangostin at 5 μg/ml (3) and the xanthones extract at 5 μg/ml (4). Matrigel invasion (c): untreated cells (1), α-mangostin at 6 μg/ml (2) xanthones extract at 6 μg/ml (3) and at 4.5 μg/ml (4).

Cell migration was also inhibited in both treatments (Figure 4b). The percentage of wound closure in the untreated cells was (65 ± 4.3)%. α-Mangostin, at 5 μg/ml, reduced the percentage of wound closure to (41 ± 2.7)%, (P = 0.0). Likewise, the xanthones extract, at 3 and 5 μg/ml, reduced the wound closure percentage to (42 ± 4.2)% and (56 ± 3.4)%, (P < 0.05). The cell invasion of matrigel was also inhibited by α-mangostin at 6 μg/ml (78 ± 6)%, and by the xanthones extract at 6 μg/ml (78 ± 8)% and 4.5 μg/ml (57 ± 8)%. Besides reducing the number of matrigel-invading cells, the treatment compounds also caused morphological changes in the treated cells characterized by cytoplasmic shrinkage and contraction of cellular polypodia (Figure 4c).

The article "In vitro and in vivo anti-colon cancer effects of Garcinia mangostana xanthones extract" was retracted in 2022. Reasons: ethical violations by an author; concerns about the data.

### Effect on cell signalling pathways

The transfected HCT 116 cells were treated at 2 concentrations 7.5 and 10 μg/ml for 6 h, and the results in the treated cells were compared to those treated with the vehicle alone (0.5% DMSO). The transcription factor activity of the 10 pathways is reduced by treating the cells with 10 μg/ml of the xanthones extract and α-mangostin. However, the treated cells showed apoptotic morphology, which indicates the downregulation of signalling pathways occurred as a consequence of apoptosis. Treatment at 7.5 μg/ml did not induce apoptotic changes in the treated cells, but resulted in differential effects on the signalling pathways. The fold changes in the transcription factor activity in cells treated at 7.5 μg/ml is displayed in Figure 5. The transcription factor activity of the MAPK/ERK pathway was increased by 71% in α-mangostin-treated cells and 97% in the xanthones extract-treated cells. Activity of the Myc/Max signalling pathway was also increased by 48% in α-mangostin and 60% in the xanthones extract-treated cells. In addition, the activity of the p53 signalling pathway was increased by 30% in α-mangostin-treated cells and 50% in the xanthones extract-treated cells. On the contrary, the activity of the NFKB pathway was inhibited by 30% in α-mangostin treatment and by 13% in the extract-treated cells. On other hand, the treatment compounds did not cause any significant changes in the Wnt, Notch, TGFB, cell cycle, hypoxia and MAPK/JNK signalling pathways.

**Figure 5:** **Effect of the xanthones extract and α-mangostin (7.5 μg/ml) on the transcription factor activity of 10 cell signalling pathways.** The fold changes in the transcription factor activity were calculated by dividing the relative light units in the treated cells by that of the untreated cells. The fold change of (1) indicates no activity.

### *In Vivo* anti-colon cancer effect

The *in vivo* anti-colon cancer effect of the xanthones extract was investigated on the HCT 116 subcutaneous tumor model established in NCR nu/nu nude mice. The results are presented as average tumor size ± SD (n = 6). The treatment with the α-mangostin extract caused apparent necrosis of the pre-established tumors in 2 animals (Figure 6a), and caused significant reduction in the tumor size compared to untreated group. Data analysis was performed by considering the tumor size on 5-days intervals and showed that significant reduction in tumor size was achieved after 15 days (0.5% wt/wt), and 20 days (0.25% wt/wt) of treatment, P < 0.05, (Figure 6b). Analysis of the tumor cross sections revealed apparent differences in the extent of necrotic regions between the treated versus untreated tumors (Figure 6c). The necrotic/apoptotic cells in treated tumors predominate over the viable tumor cells which appear as islands in the middle of necrotic cells. On the contrary, untreated tumors were more compact with more abundance of viable tumor cells.

The article "In vitro and in vivo anti-colon cancer effects of Garcinia mangostana xanthones extract" was retracted in 2022. Reasons: ethical violations by an author; concerns about the data.

**Figure 6:** **The subcutaneous tumors in NCR nude mice (a): Untreated group (1), and the treated group at 0.5% wt/wt of the xanthones extract (2).** Analysis of tumor size (b): analysis of tumor size versus time (days) after treatment with the xanthones extract at 2 doses 0.5% and 0.25% wt/wt compared to the control group (untreated). (*) refers to significant difference between both treated groups (P < 0.05) and the control, and (#) refers to significant difference between the 0.5% group and the control in each corresponding interval. Cross sections of tumor tissues (c): untreated animals (1), 0.5% treated group (2) and the 0.25% treated group (3). The tissues were stained with Hematoxylin-eosin and the pictures were captured at 5× magnification. (N) refers to necrotic cells and (V) refers to viable tumor cells.

The average number of intratumor blood vessels was 3.9 ± 0.6/microscopic field (0.5% wt/wt) and 4 ± 0.3/microscopic field (0.25% wt/wt), was significantly lower than that in the control group (7.8 ± 1.2), P = 0.0.

Additionally, effect on the animal body weight was also investigated and the results are presented as average percentage of weight gain or loss. The data showed a slight, but not statistically significant weight loss in the treated groups −4.4 ± 10% (0.5% wt/wt) and −1.5 ± 2.4% (0.25% wt/wt), compared to 5.3 ± 6% (control group), P = 0.1 and 0.4, respectively.

## Discussion

The xanthones extract of *G. mangostana* fruit rinds contains mainly α-mangostin and γ-mangostin. The HCT 116 cell line was selected as a model of human colorectal carcinoma [33], and CCD-18Co human normal fibroblast was selected as a control cell line. The cytotoxicity of the xanthones extract, α-mangostin and γ-mangostin was comparable to that of cisplatin, and the xanthones extract was almost 2 times more cytotoxic on the colon cancer cells than on the normal cells, which indicates higher selectivity towards the colon cancer cells.

Apoptosis studies revealed enhancement of the executioner caspases-3/7, activation of the initiator caspase-9, induction of DNA fragmentation and chromatin condensation, and loss of mitochondrial membrane potential. These results indicate the role of the mitochondrial pathway of apoptosis in mediating cytotoxicity of the compounds. Our results are consistent with the previous results of other researchers [10,34], and provide further evidence on apoptotic effects of *G. mangostana*, and indicate the xanthones of this fruit as potential anti-cancer candidates.

The article "In vitro and in vivo anti-colon cancer effects of Garcinia mangostana xanthones extract" was retracted in 2022. Reasons: ethical violations by an author; concerns about the data.

Sub-cytotoxic concentrations of α-mangostin and the xanthones extract inhibited 3 key steps in tumor metastasis including the cell migration, cell invasion and clonogenicity. These results, in combination the results of other researchers [9,35], indicate the potential anti-metastatic effect of the *G. mangostana* xanthones.

In order to gain deeper insights into the mechanism of action, a cell-based reporter assay was used to study the effect of α-mangostin and the xanthones extract on the transcription factor activity of the Notch, Wnt/β-Catenin, TGFβ, p53, HIF, Myc, E2F, NFKB, MAPK/ERK (SRE), and MAPK/JNK (AP-1) signalling pathways. The compounds enhanced the transcription factor activity of the MAPK/ERK, Myc/Max, and p53/DNA damage signalling pathways. Previous research showed that the activated ERK pathway is associated with increased stability and activity of p53, and increased stability of c-Myc that in turn increases the proapoptotic effects of p53 tumor suppressor gene [36,37]. Recent studies showed that activation of the ERK pathway is implicated in inducing apoptosis, as a consequence of DNA damage caused by cisplatin [38], etoposide [39], doxorubicin, and ionizing and Ultraviolet irradiation [40]. Therefore, upregulation of the ERK pathway may provide a therapeutic target for different types of cancer [41-43], however further investigation is required to study the effect of the activated ERK pathway on the expression of the proapoptotic proteins such as p21 and Bax. α-Mangostin also caused inhibition of the NFKB pathway. The downregulation of this pathway is associated with increased sensitivity of chemoresistant cells [44], and hence α-mangostin may sensitize the colon cancer cells to the apoptotic effect of chemotherapeutics.

Different mechanisms of action of mangostins have been reported including upregulation of the ERK ½ in DLD-1 colon cancer cells [8], inhibition of TCF/β-catenin transcriptional activity in colon cancer cells [11], and inhibition of the MAPK/ERK, MAPK/JNK and Akt signalling pathways in human chondrosarcoma cells [45]. These findings indicate that mangostins may work by different mechanisms in different tumor cells. Drug concentration and duration of treatment have significant effects on viability of cells, and hence these may have substantial effect on the activity of signalling pathways.

The *In vivo* anti-colon cancer study revealed significant inhibition of the tumor growth. The Anti-tumor effect of the extract may be explained due to direct cytotoxicity on the tumor cells as evident by the presence of extensive necrosis in the subcutaneous tumors, or due to reducing the intratumor blood supply as evident by the significant reduction in the number of intratumor blood vessels, or due to combination of both mechanisms.

The article "In vitro and in vivo anti-colon cancer effects of Garcinia mangostana xanthones extract" was retracted in 2022. Reasons: ethical violations by an author; concerns about the data.

## Conclusions

Taken together, our data suggest new mechanisms of action of α-mangostin and suggest the xanthones extract of *G. mangostana* as a potential anti-colon cancer candidate.

## Competing interests

The authors declare no conflict of interest related to this work.

## Authors’ contributions

AFA carried out the experiments, performed the statistical analysis, and drafted the manuscript. KM interpreted the results of cell signalling pathways and helped in editing the manuscript. ZI interpreted the LC-MS data. AMS participated in the design of the study and edited the manuscript. All authors read and approved the final manuscript.

## Pre-publication history

The pre-publication history for this paper can be accessed here:

http://www.biomedcentral.com/1472-6882/12/104/prepub
